The article "Machine Learning-Based Gynecologic Tumor Diagnosis and Its Postoperative Incisional Infection Influence Factor Analysis" was retracted in 2023. Reasons: signs of a paper mill; compromised peer review; unreliable results or conclusions.

# Machine Learning-Based Gynecologic Tumor Diagnosis and Its Postoperative Incisional Infection Influence Factor Analysis

**DOI:** 10.1155/2021/7956184

**Published:** 2021-11-23

**Authors:** Qian Shen, Ling Wang

**Affiliations:** ^1^Department of Surgical Anesthesiology, Huangshi Central Hospital, Huangshi 435000, China; ^2^Department of Obstetrics and Gynaecology, Huangshi Central Hospital, Huangshi 435000, China

## Abstract

Various factors influencing postoperative incisional infection in gynecologic tumors were analyzed, and the value of quality nursing intervention was studied. In this study, 74 surgically treated gynecologic tumor patients were randomly selected from within the hospital as the study population and were divided into study and control groups. For this purpose, the whole-group random sampling method is utilized to compare the postoperative incisional infection rates of the two groups, analyze their influencing factors, and develop quality nursing interventions. In this paper, a breast cancer diagnosis prediction model was developed by combining the self-attentive mechanism. The preprocessing work such as data quantification and normalization was performed first which is followed by adding the preprocessed data to the self-attentive mechanism. This model has solved the problem that recurrent neural networks (RNNs) could not extract and calculate the features at the same time. Likewise, it has solved the drawback that the RNN could not consider global features at the same time when extracting the features, and then, the feature matrix extracted by the self-attentive mechanism was added to the adaptive neural network. The adaptive neural network model for breast cancer diagnosis prediction was constructed and, finally, relevant parameters of the adaptive neural network model were adjusted according to different tasks to make the model performance optimal. Experimental results showed that the postoperative incision infection rate of patients in the study group was 2.70%, which was significantly lower than that of 21.62% in the control group (*P* < 0.05). Likewise, operation time, operation method, hospitalization time, preoperative fever, diabetes mellitus, and anemia were the main influencing factors of postoperative incision infection in women with gynecologic tumors. The time of surgery, surgical method, long hospital stay, preoperative fever, diabetes, and anemia are the main factors that lead to postoperative incisional infection in female gynecologic tumor patients.

## 1. Introduction

Gynecologic tumor is a common gynecologic disease, which poses serious danger to women's physical and mental health, and one of the most common clinical treatment methods is surgery. Therefore, if postoperative incision infection occurs in female gynecologic tumor patients, it will not only affect the treatment effect and increase the treatment burden of patients but also lead to the failure of surgery [1]. Therefore, it is important to analyze the factors affecting postoperative incisional infection in female gynecologic tumor patients and then develop a targeted quality nursing intervention program to improve the effect of female gynecologic tumor surgical treatment. Based on this, this study randomly selected 74 female gynecologic tumor patients treated surgically and analyzed the clinical treatment effect of quality nursing care.

The article "Machine Learning-Based Gynecologic Tumor Diagnosis and Its Postoperative Incisional Infection Influence Factor Analysis" was retracted in 2023. Reasons: signs of a paper mill; compromised peer review; unreliable results or conclusions.

Health is the basis of comprehensive human development, and with the continuous improvement of human life quality, health conditions are gradually being paid attention to. With the advent of the era of big data, people have gradually started to focus on applying the existing artificial intelligence technology reasonably and effectively in medical research and the construction of medical informatization has become an important national development strategy [1]. The medical industry is complex and varied, which contains many aspects, such as registration, imaging, testing, diagnosis, and medication, which makes patients spend a lot of time and energy on disease prevention and treatment and also brings great challenges to the work of doctors. In traditional medical treatment, doctors make diagnosis and clinical decisions of diseases based on patients' symptoms combined with their professional knowledge and clinical experience accumulated over the years and doctors may make subjective errors in judgment. In addition, many patients in remote areas cannot receive good treatment due to the lack of medical resources and many people miss the best time to treat their diseases due to untimely access to medical care.

In traditional medical diagnostic studies, physicians use common data analysis software (e.g., SPSS and STAT) for simple analysis of clinical text data or medical image data. This software is usually based on statistical methods and does not really explore the hidden correlations or causal relationships between symptoms and diseases in the data. The application of machine learning methods in the medical field has solved the difficulties in the process of patient consultation, disease treatment, and doctor's diagnosis and decision making, and both patients and doctors can benefit from it. The processing of medical structured and unstructured data through machine learning algorithms helps to accurately analyze patients' conditions, assist doctors in making more accurate diagnoses, and improve work efficiency.

The article "Machine Learning-Based Gynecologic Tumor Diagnosis and Its Postoperative Incisional Infection Influence Factor Analysis" was retracted in 2023. Reasons: signs of a paper mill; compromised peer review; unreliable results or conclusions.

Among the most common diseases in women, breast-related diseases are particularly prominent, mainly including mastitis, breast enlargement, breast cysts, and breast cancer, the most serious of which is breast cancer (BC). A survey in the United States showed that more than 1.6 million people suffered from cancer and about 600,000 cancer deaths in 2016, among which breast cancer is the main cancer death disease among young and middle-aged women [2]. In recent years, the probability rate of women diagnosed with breast cancer in China has increased more than that in developed countries, which is extremely affecting health. In 2009, the All-China Women's Federation and the National Health Care Commission started to actively implement and promote a national screening program for rural women for “two cancers,” which was fully implemented in 2016 to help women raise awareness of health care and prevention and reduce the incidence of breast cancer [3]. While it is difficult for doctors to determine the severity of a patient's disease based on complex data of breast characteristics when diagnosing breast diseases, computer technology allows the available data to be analyzed, predicted, and quickly output the disease. At the same time, the diagnosis of the disease varies from patient to patient in terms of signs and symptoms and doctors need to make a diagnosis based on the signs and symptoms of different patients combined with pathological data. The feature data generated in this process are complex and variable, and doctors will make judgments by combining their previous medical experience, so different doctors may give different diagnosis results. To solve this problem, this paper proposes two breast cancer disease diagnosis prediction models based on deep learning models and integrated learning models to help doctors improve efficiency and reduce workload.

In this paper, traditional machine learning algorithms were used to assist patients or doctors to make preliminary diagnosis based on relevant symptoms exhibited by patients. This system helps patients decide whether they should go to breast cancer-related departments for consultation. Likewise, it analyzes relevant pathological data of patients, particularly after admission which is based on deep learning models and integrated learning models, to build a breast cancer disease diagnosis prediction model to assist doctors to carry out clinical related work.

In the subsequent section, a brief literature review or study is presented. A proposed model is described, which is followed by various dataset descriptions utilized in this study. In Section 4, general information and guidelines about the proposed mechanism are presented. Finally, concluding remarks are given, along with future directives.

The article "Machine Learning-Based Gynecologic Tumor Diagnosis and Its Postoperative Incisional Infection Influence Factor Analysis" was retracted in 2023. Reasons: signs of a paper mill; compromised peer review; unreliable results or conclusions.

## 2. Literature Review

The rapid development of data mining techniques such as machine learning and deep learning has led to the widespread use of data analysis techniques, enabling knowledge discovery to progress both horizontally and vertically. Currently, machine learning has achieved some results in healthcare-related fields. Combined with the research conducted in this paper, this section will briefly introduce the existing research work from the following two aspects: In the medical profession, a series of abnormal changes that occur in a patient's body are referred to as clinical manifestations of a patient suffering from a certain disease. Clinical manifestations are divided into symptoms and signs. Symptoms include cough, fever, weakness of the limbs, and others. A single disease usually has multiple symptoms, and many diseases present with the same symptoms. Usually, researchers classify symptoms by the location of the symptoms, the nature of the symptoms, the role of the symptoms in identification, and the clinical department classification.

The behavioral symptoms caused by Parkinson's disease were continuously monitored, and a support vector machine (SVM) model was used to identify the symptoms of motor retardation in Parkinson's disease, achieving a high classification accuracy [4]. The EEG data of female participants suffering from depression were classified using random forest and support vector machine, which in turn assessed the neurophysiological characteristics of this group of patients. CNN and question-and-answer models were combined to classify skin symptoms and thus make better decisions about treatment [5]. Hartmann et al. monitored symptom changes and used a longitudinal clustering algorithm to classify symptoms in order to better evaluate the treatment of depression [6].

A context-independent grammar approach was used to improve the accuracy of the original classification of symptoms using the classification and regression trees (CART) algorithm by 5% [7]. A thorough analysis of the clinical characteristics and admission departments of patients with ovarian epithelial tumors using a large sample of data found a correlation between clinical characteristics and admission departments [8].

Word vector and BP models were applied to classify and extract data from electronic health records to solve the problem of automatic categorization of symptom information in medical records, with a model accuracy of 71.7% [9]. A Bayesian algorithm was used to mine the relationship between symptoms and symptoms in TCM to adjust prescriptions [10]. A model based on high-dimensional attribute similarity calculation was proposed to classify symptoms by analyzing data associated with symptoms (e.g., drugs and prescriptions) [11]. An integrated learning (MPEL) algorithm, which is based on a multimodal perturbation strategy, was proposed to train the “symptom-certification” case data of TCM asthma, and the model performed well in classification prediction with high accuracy [12]. A statistical study was conducted on the first symptoms of ANCA-associated small vessel vasculitis and the departments visited and pointed out that the first symptoms of this disease are diverse and the departments visited are scattered [13].

The article "Machine Learning-Based Gynecologic Tumor Diagnosis and Its Postoperative Incisional Infection Influence Factor Analysis" was retracted in 2023. Reasons: signs of a paper mill; compromised peer review; unreliable results or conclusions.

The clinical manifestations of patients often play a crucial role in the diagnosis of diseases, and researchers study medical symptoms through machine learning methods or deep learning methods to assist doctors to work more accurately and efficiently, improving the quality and efficiency of their work.

Based on the abovementioned existing studies, it is easy to see that most of the current studies on disease symptom classification use machine learning methods to find associations between symptoms and specific diseases. Although authors have found some correlation between the clinical characteristics of patients with ovarian epithelial tumors and the department in which they were admitted; instead, a statistical approach was used to develop the study [11].

The introduction of “precision medicine” has led to the rapid development of the “Internet medicine” model, and the role of clinical disease diagnosis and prediction models in medical diagnosis and treatment decisions, patient prognosis management, and public health resource allocation has become increasingly prominent. Traditional machine learning and deep learning models use historical data and real-time data to quickly analyze and produce results. By building diagnostic predictive models for diseases, they can assist doctors in making better decisions about patients. By building a predictive model for disease diagnosis, it can assist doctors in making better decisions about patients' conditions and thus improve medical care. The model building process is shown in Figure 1.

The presence of malignant cells in breast cancer was predicted using logistic regression (LR), SVM, and random forest (RF) models based on blood sample data, where the sensitivity of using SVM ranged from 82% to 88%. A combination of migration learning and CNN was used for breast cancer cell detection and cancer cell classification with a model accuracy of more than 97%. An evolutionary algorithm-based Memetic Pareto Artificial Neural Network (MPANN) method was proposed for breast cancer prediction, which resulted in a higher standard deviation of test accuracy than the reduced 0.459. The evolutionary algorithm NSGA-III (nondominated sorting genetic algorithm-III) was proposed to initialize a deep neural network (DNN) and tune the network as a judgment of the outcome of breast cancer disease treatment.

The article "Machine Learning-Based Gynecologic Tumor Diagnosis and Its Postoperative Incisional Infection Influence Factor Analysis" was retracted in 2023. Reasons: signs of a paper mill; compromised peer review; unreliable results or conclusions.

A genetic algorithm-based online gradient boosting (GAOGB) model was proposed for breast cancer diagnosis and prognostic guidance instructions through online learning techniques at any time. An end-to-end deep learning system that combines Full Convolutional Network (FCN) was proposed to extract breast region data, and the results have a high correlation with the diagnosis made by pathologists.

Researchers use traditional machine learning algorithms or deep learning algorithms to integrate medical books and medical records, and clinical researchers use traditional machine learning algorithms or deep learning algorithms to integrate medical books, medical records, clinical treatment records, experimental data, and other information to provide patients with medical treatment recommendations. It is easy to see that data mining has been fully introduced into the clinical medical field, providing reference for doctors to make diagnosis and quickly develop effective treatment plans. It is easy to see that data mining has come into the clinical medical field to provide a reference for doctors to make diagnosis and quickly develop effective treatment plans. Diagnosis and prediction of diseases will serve as the basis for the refinement of the medical industry. Diagnostic and predictive research will provide a strong theoretical basis for the refinement of medical services.

Researchers have built many disease diagnosis prediction models using machine learning methods, among which a number of studies have been conducted on different breast cancer data, but there is no multitask breast cancer disease diagnostic. The construction of multitask breast cancer disease diagnosis prediction models has not been conducted.

## 3. Proposed Model

In recent years, deep learning has widely been used in the medical field and among various deep learning algorithms, the introduction of an attention mechanism makes the proposed algorithm purposely focus on some more critical input information and process it during the execution, which greatly improves the efficiency of neural networks. In this paper, we propose an adaptive deep learning model with the introduction of a self-attention mechanism for breast cancer diagnosis prediction research.

### 3.1. Method Construction Process

The construction of our method starts with data acquisition and then data preprocessing, followed by the introduction of the self-attentive mechanism into the neural network, the combination of the self-attentive mechanism and the neural network for the training of the adaptive model, by which the model can find the best adaptive model according to different tasks, and finally, the validation of the model. The model construction process can be divided into four parts as in Figure 2:

1. *Data Collection*. In this paper, two publicly available breast cancer datasets from the University of California UCI database were used to train and test the model. The datasets specifically include the breast cancer diagnosis dataset and the breast cancer recurrence dataset.
2. *Data Preprocessing*. The data are first quantified, and then, the missing values are processed to ensure high-quality data in the input model.
3. *Training Model*. During the training process, the adaptive network is adjusted according to the different datasets to achieve the optimal training model.
4. *Model Validation*. The selected test set data are compared with the experimental results of the prediction model, and multiple evaluation index pairs are used to evaluate.

The article "Machine Learning-Based Gynecologic Tumor Diagnosis and Its Postoperative Incisional Infection Influence Factor Analysis" was retracted in 2023. Reasons: signs of a paper mill; compromised peer review; unreliable results or conclusions.

### 3.2. Data Preprocessing Techniques

Data preprocessing is one of the most fundamental and important aspects of machine learning. Usually, the data determine how well the model works, and the algorithm is only an infinite approximation to the optimal result. In the study described in this paper, since the data needed to build the model are no longer text data, natural language processing is not required. For the characteristics of the data in the section of this paper, data preprocessing techniques of data transformation and data cleaning are mainly used to ensure the high quality of the data input to the breast cancer diagnosis prediction model.

#### 3.2.1. Data Introduction

The source data for this paper on breast cancer disease diagnosis prediction model construction are two types of breast cancer pathology datasets from the University of California UCI database (https://archive.ics.uci.edu/ml/datasets.php), namely, the breast cancer diagnosis characteristics dataset (DataSet1) and the breast cancer recurrence characteristics dataset (DataSet2). In this paper, the proposed two models will be trained and measured using these two datasets. The DataSet1 dataset contains 9 features, and the DataSet2 dataset has 9 features, and the features of the dataset include numerical and categorical data.

In the DataSet1 dataset, the features include the thickness of the mass, the size of the tumor cells, the shape of the tumor cells, the number of chromosomes, the location of the mass, and other attributes, and the data features are all numerical in nature.

The article "Machine Learning-Based Gynecologic Tumor Diagnosis and Its Postoperative Incisional Infection Influence Factor Analysis" was retracted in 2023. Reasons: signs of a paper mill; compromised peer review; unreliable results or conclusions.

In the DataSet2 dataset, features include attributes such as patient's age, menopause status, tumor size, tumor shape, and the presence of nodules. Each feature dataset contains numeric data and textual data.

#### 3.2.2. Data Preprocessing

The original text dataset is first imported into the database, and the features are quantified using SQL statements. Then, the missing values were filled using the mean value method. In the experiment, it was found that the records that could not be filled were fewer and had less impact on the whole dataset, so the records that could not be filled were discarded.

### 3.3. Attentional Mechanisms

The attention mechanism (AM) model was proposed by the Google team in 2014. The main idea, which mimics human attenton, is to focus limited energy and attention on what is important. It is to selectively filter out the more relevant and close information from the huge amount of information. The importance of information mainly depends on the application scenario, and attention is divided into two types according to the application scenario: one for processing image data, called spatial attention, and the other for natural language processing, called temporal attention. Currently, most attention models rely mainly on the encoder-decoder (Encoder-Decoder) framework [14], as shown in Figure 3, and are mainly applied to the seq2seq problem.

The encoder-decoder process is divided into two parts: the encoder process is to encode the input sentence to form the intermediate semantic code C, and the decoder process is to decide to select the word with the highest probability to form the sentence based on the semantic code C and the word output above [4].

The attention model is based on the encoder-decoder framework, and the weight of a word is determined by the different roles of the word in the semantics. In the encoder process, the input is no longer the semantic code C, but a sequence of different semantic codes which is shown in Figure 4.

The encoding-decoding framework in natural language processing can be understood as a process in which one sentence generates another sentence; the encoder process is responsible for learning the semantic encoding C from the input sentence, and the decoder process generates the target sentence with reference to the semantic encoding C [14]. Combining encoder-decoder with the attention mechanism would be to adapt the previously fixed C to vary according to the current output words *C*_*i*_, where each *C*_*i*_ corresponds to the weight assigned to the attention of the words in the original utterance.

The article "Machine Learning-Based Gynecologic Tumor Diagnosis and Its Postoperative Incisional Infection Influence Factor Analysis" was retracted in 2023. Reasons: signs of a paper mill; compromised peer review; unreliable results or conclusions.

### 3.4. Method Implementation

In traditional machine learning techniques, the features that describe a sample are usually determined by experts. The advent of neural networks has enabled machines to mimic human thinking and visual and auditory activities and to learn more autonomously and automatically how to learn and process features.

In this paper, in the process of constructing our method, we not only introduce the self-attentive mechanism but also combine it with neural networks to build adaptive neural networks so that the model can adjust its relevant parameters according to different tasks and thus achieve the optimal prediction accuracy under different tasks. The core of the self-attentive mechanism is shown in the following equation:

(1) $$\begin{array}{c} \alpha_{i,j}=\frac{q^{i}\cdot k^{j}}{\sqrt{d}}, \end{array}$$

where *q* stands for query (to match others), *k* stands for key (to be matched), and *d* denotes the dimension of *q* and *k* dim.

The breast cancer diagnosis prediction model based on our method is described in Algorithm 1.

In this paper, a self-attentive mechanism is introduced into the adaptive neural network so that the model focuses on the more important feature information during the training process. From the internal structure of the model, the self-attentive mechanism can associate its own features with all the features before and after them when processing the features, solving the problem that RNN cannot parallelize operations and the problem that CNN can only convolve local features at a time and cannot consider global features when processing features is also solved. Our approach is shown in Figure 5.

### 3.5. Evaluation Indicators

Evaluation metrics are important criteria for assessing how well a machine learning model works for the task that has been performed, and this step assesses the effectiveness and performance of the algorithms used. Usually, researchers choose relevant evaluation metrics depending on the machine learning task. The evaluation metrics that are commonly used in classification tasks are commonly used evaluation metrics for classification tasks [6] such as accuracy, precision, recall, F1-score, and ROC curve.

The confusion matrix is a matrix used to describe the classification performance of a classification model based on the number of predicted and true samples. Assuming that the binary classification task contains two classes, 0 and 1, the distribution of the confusion matrix can be divided into the following four ways:

  TPs (True Positives): the actual value of the sample is 1, and the predicted value of the model is 1
  TNs (True Negatives): the actual value of the sample is 0, and the predicted value of the model is 0
  FPs (False Positives): the actual value of the sample is 0, and the predicted value of the model is 1
  FNs (False Negatives): the actual value of the sample is 1, and the predicted value of the model is 0

The confusion matrix is shown in Table 1.

The article "Machine Learning-Based Gynecologic Tumor Diagnosis and Its Postoperative Incisional Infection Influence Factor Analysis" was retracted in 2023. Reasons: signs of a paper mill; compromised peer review; unreliable results or conclusions.

#### 3.5.1. Accuracy

The accuracy rate is calculated as the percentage of correctly classified samples out of the total samples in the results of the model run. The accuracy rate aims to indicate the accuracy of the model's prediction results for positive and negative samples as a whole, as shown in the following equation:

(2) $$\begin{array}{c} \text{accuracy}=\frac{TP+TN}{TP+FN+FP+TN}. \end{array}$$

#### 3.5.2. Precision

The precision rate is from the perspective of prediction results, i.e., the rate of no misspecification. The precision rate aims to illustrate the accuracy of the model's prediction results for positive samples, as shown in the following equation:

(3) $$\begin{array}{c} \text{precision }=\frac{TP}{TP+FP}. \end{array}$$

#### 3.5.3. Recall

The recall rate, on the other hand, is for the original sample data set and indicates the percentage of the original positive samples that are accurately classified as positive samples. The calculation formula is given in the following equation:

(4) $$\begin{array}{c} \text{recall }=\frac{TP}{TP+FN}. \end{array}$$

#### 3.5.4. F1-Score

The F1 value depends on the precision rate and recall rate and defines the summed mean value of both the precision rate and recall rate. The formula is defined in the following equation:

(5) $$\begin{array}{c} \;F1=\frac{2TP}{2TP+FP+FN}. \end{array}$$

#### 3.5.5. ROC Curve

The ROC curve is an evaluation method introduced specifically for the medical field [7]. The horizontal coordinate of the two-dimensional curve is the false positive rate [8] (FP_rate), i.e., the number of actual negative samples that the model incorrectly predicts to be positive as a percentage of the original negative samples; the vertical coordinate of the two-dimensional curve is the true rate (TP_rate), i.e., the number of actual positive samples that the model predicts to be positive as a percentage of the original positive samples. The formulas for calculating the horizontal and vertical coordinates of the ROC curve (i.e., false positive rate and true rate) are given in the following equations:

(6) $$\begin{array}{c} FP\_\text{rate}=\frac{FP}{FP+TN}, \end{array}$$

(7) $$\begin{array}{c} TP\text{\_rate}=\frac{TP}{TP+FN}. \end{array}$$

The ROC curve must pass through the points (0, 0) and (1, 1) for the model effect. The closer the curve is to the point (0, 1), the better the model effect; i.e., the higher the true rate, the better the effect. This essentially shows the change of the recall rate of a model under different threshold values, which is shown in Figure 6.

The article "Machine Learning-Based Gynecologic Tumor Diagnosis and Its Postoperative Incisional Infection Influence Factor Analysis" was retracted in 2023. Reasons: signs of a paper mill; compromised peer review; unreliable results or conclusions.

### 3.6. Experimental Results

During the experiments, 70% of the breast cancer pathology data were selected as the training set and 30% of the data were selected as the test set for each data set. The experiments in this paper consist of two parts:

1. Adjust the relevant parameters of the adaptive neural network model according to different datasets and select the best adaptive neural network model
2. Compare the experimental results of our method with those of RNN, CNN, and long and LSTM

#### 3.6.1. Parameter Selection of Adaptive Neural Networks

In this paper, the two datasets are added to the self-attentive mechanism algorithm. Then, the feature matrix obtained from the self-attentive mechanism is added to the adaptive neural network, and then, the grid search method is used to tune the neural network. In this paper, we add the two datasets to the self-attentive mechanism algorithm and then add the feature matrix obtained from the self-attentive mechanism to the adaptive neural network. In the selection of the adaptive neural network using the grid search method for the DataSet1 dataset, the model is trained mainly for the layer and shape parameters with stddev = 0.1.

It was found that the accuracy of the prediction model based on our method was maintained at 65.4% when the layer of the adaptive neural network model was ≤ 3 during the training of the breast cancer diagnosis task (DataSet1 dataset). According to the experimental results shown in Table 2, the accuracy of the adaptive neural network model gradually increases as the number of neurons in the layer and shape of the model increases; however, the accuracy of the adaptive neural network model does not increase when the number of neurons in the layer and shape of the adaptive neural network model increases to a certain number.

In summary, when the DataSet1 dataset was used as input for the breast cancer diagnosis task, the prediction model based on our method with the selected adaptive neural network model with parameter layer = 4, shape = {[8,400], [400,200],][200,50],[50,2]}, and stddev = 0.1 worked best. The model has the best accuracy of up to 99%.

For the breast cancer recurrence prediction task (DataSet2 dataset), the parameters of the adaptive neural network are still selected using the grid search method and the models corresponding to the layer and shape parameters are trained for stddev = 0.1 and stddev = 1, respectively. For the DataSet2 dataset, the results of the adaptive neural network models with different parameters are shown in Table 2.

The article "Machine Learning-Based Gynecologic Tumor Diagnosis and Its Postoperative Incisional Infection Influence Factor Analysis" was retracted in 2023. Reasons: signs of a paper mill; compromised peer review; unreliable results or conclusions.

As the layer and shape of the adaptive neural network model are expanded, the prediction accuracy of the model increases; however, when the layer and shape of the model are increased to a certain number, the accuracy of the model does not improve accordingly, and it is found that the accuracy of the model when stddev = 0.1 is not lower than that of the model when stddev = 1, while the other two parameters of the adaptive neural network are kept constant. The accuracy of the model with stddev = 0.1 is not lower than that with stddev = 1. The results of the relevant parameters and the corresponding model accuracy are shown in Figure 7.

In summary, when the DataSet2 dataset is used as input for the recurrence prediction task analysis, the accuracy of the model is optimal when layer = 4 or layer = 5 with stddev = 0.1 and shape = {[5,400], [400,200], [200,50], and [50,2]}. Considering the efficiency of the model operation, the parameters of the adaptive neural network model were finally selected as layer = 4, stddev = 0.1, and shape = {[5,400], [400,200], [200,50], and [50,2]}. With this parameter, the prediction accuracy of the adaptive neural network model can reach 88.7%.

#### 3.6.2. Comparison of Experimental Results

The experimental results of our method are compared with those of RNN, CNN, and LSTM. The experimental results are shown in Tables 2 and 3, respectively.

As shown in Table 2, the model evaluation metrics such as accuracy, precision, and recall of the adaptive neural network model proposed in this paper in the DataSet1 dataset show good experimental results. The model ROC curves are shown in Figure 8.

As shown in Table 3, with the DataSet2 dataset, the accuracy and recall of the breast cancer diagnosis prediction model based on our method proposed in this paper obtained better experimental results in terms of evaluation metrics. The accuracy rate of the model reaches 88.7%. The accuracy comparison of the experiments is shown in Figure 9.

## 4. Information and Discussion

### 4.1. General Information

In this study, 74 female gynecologic tumor patients admitted for surgical treatment were randomly selected within the hospital as study subjects, and with the patients' informed consent, they were divided into study and control groups using the whole-group random sampling method. There were 37 patients in the study group, aged 60–78 years, with an average age of 67.52 ± 2.06 years. Among them, there were 11 patients with cervical cancer, 13 patients with uterine fibroids, 8 patients with ovarian tumors, and 5 patients with endometrial cancer. There were 16 patients with laparoscopic surgery and 21 patients with open surgery. There were 37 patients in the control group, aged 61–77 years, with an average age of 65.19 ± 1.08 years. Among them, there were 9 patients with cervical cancer, 10 patients with uterine fibroids, 11 patients with ovarian tumors, and 7 patients with endometrial cancer. There were 19 patients with laparoscopic surgery and 18 patients with open surgery. The basic data of the two groups were statistically processed, with *P* > 0.05, no statistical difference, comparable.

The article "Machine Learning-Based Gynecologic Tumor Diagnosis and Its Postoperative Incisional Infection Influence Factor Analysis" was retracted in 2023. Reasons: signs of a paper mill; compromised peer review; unreliable results or conclusions.

### 4.2. Results

Comparing the postoperative incision infection rates of the two groups, it can be seen from Table 1 that the postoperative incision infection rate of patients in the study group was 2.70%, which was significantly lower than that of the control group, 21.62%, and the difference was statistically significant, *P* < 0.05, which is shown in Table 4.

The multifactorial, logistic regression analysis of the factors affecting postoperative incisional infection in the two groups of patients showed that the time of surgery, surgical method, length of hospital stay, preoperative fever, diabetes mellitus, and anemia were the main factors affecting postoperative incisional infection in women with gynecologic tumors, as shown in Table 5.

## 5. Discussion

Gynecologic tumors are a major threat to women's health, and with the increasing trend of female gynecologic tumor patients in recent years, it seriously affects the lives and health of women. The common treatment for gynecologic tumors is surgical resection, but this type of surgery, especially for malignant tumors, is not only longer and more complicated but also involves many organs, which usually causes great trauma to patients, and most women are immunocompromised, so they are prone to postoperative incisional infections and other common complications [2]. Once incisional infection occurs, it will not only affect the patient's treatment outcome but also increase the patient's pain and, in severe cases, may even induce systemic inflammatory reactions, leading to surgical failure. Therefore, it is important to analyze the factors influencing postoperative incisional infection in gynecologic tumors in the elderly in order to prevent infection. In this study, it was found that time of surgery, surgical approach, hospitalization, preoperative fever, diabetes, and anemia were the main factors influencing postoperative incisional infections in gynecologic tumors. Prevention of postoperative incisional infections is not only related to clinical procedures and medications but also nursing interventions play an important role [3]. The main reason for this is that the implementation of quality nursing interventions has increased the intensity and improved the quality of daily inspections by medical and nursing staff, which is of great value in the predictive assessment of infection in patients.

The article "Machine Learning-Based Gynecologic Tumor Diagnosis and Its Postoperative Incisional Infection Influence Factor Analysis" was retracted in 2023. Reasons: signs of a paper mill; compromised peer review; unreliable results or conclusions.

The results of this study showed that the rate of postoperative incisional infection in the study group was 2.70%, which was significantly lower than that in the control group, which was 21.62% (*P* < 0.05); time of surgery, surgical approach, length of hospital stay, preoperative fever, diabetes, and anemia were the main factors influencing postoperative incisional infection in elderly gynecologic oncology patients. In conclusion, the time of surgery, surgical method, prolonged hospital stay, preoperative fever, and the presence of diabetes and anemia are the main factors leading to postoperative incisional infections in female gynecologic oncology patients, and quality nursing interventions have better clinical care effects in preventing postoperative incisional infections and should be widely used in clinical care.

## 6. Conclusion

In this paper, a breast cancer diagnosis prediction model is constructed by combining the self-attentive mechanism. Initially, data are quantified and normalized. Then, we add the preprocessed data into the self-attentive mechanism and then add the feature matrix extracted by the self-attentive mechanism into the adaptive neural network to build the adaptive breast cancer diagnosis prediction neural network model. The experimental results show that the dataset used in this paper has a good experimental effect on the breast cancer diagnosis prediction model based on our method. A very important consideration for deep learning versus traditional machine learning is the size of the sample. Generally speaking, the deep learning ability or fitting ability of the model in deep learning is significantly stronger than that of traditional machine learning models, so a large amount of data is required for training to ensure the stability of the model. Therefore, in this paper, after constructing a breast cancer diagnosis and prediction model using deep learning, we propose the use of a large amount of data for training. Therefore, after using deep learning to build a breast cancer diagnosis prediction model, we have proposed the use of an integrated learning model which is based on machine learning to build a breast cancer diagnosis prediction model.

In the future, we will try to expand the operational capabilities of the proposed model for other commonly known diseases. In addition, we are trying to expand the proposed methods by integrating them with existing models.

## Figures and Tables

**Figure 1:** Process of building a predictive model for disease diagnosis.

The article "Machine Learning-Based Gynecologic Tumor Diagnosis and Its Postoperative Incisional Infection Influence Factor Analysis" was retracted in 2023. Reasons: signs of a paper mill; compromised peer review; unreliable results or conclusions.

**Figure 2:** Diagram of the construction process of the proposed method.

**Figure 3:** Encoder-decoder framework diagram.

**Figure 4:** Attention's schematic.

**Figure 5:** Diagram of the proposed approach.

**Figure 6:** ROC curve.

**Figure 7:** Adaptive neural network parameter selection.

**Figure 8:** ROC curve (Dataset1).

**Figure 9:** Model accuracy comparison.

**Algorithm 1:** The proposed algorithm.

**Table 1:** Confusion matrix.

Actual value/estimate	1	0
1	TP	FN
2	FP	TN

**Table 2:** Comparison of model accuracy, precision, recall, and F1 values (DataSet1).

	RNN	CNN	LSTM	Our method
Accuracy	0.985	0.99	0.985	0.99
Precise	0.993	0.985	0.993	0.993
Recall	0.993	1.0	0.993	0.993
F1	0.989	0.993	0.989	0.993

**Table 3:** Comparison of model accuracy, recall, and F1 values (DataSet2).

	RNN	CNN	LSTM	Our method
Precise	1.0	0.868	0.868	0.884
Recall	0.924	0.967	0.967	1.0
F1	0.895	0.915	0.924	

**Table 4:** Comparison of postoperative incisional infection rates between two groups of patients.

Group	N	Number of infections (*n*)	Infection rate (%)
Research group	37	1	2.70
Control group	37	8	21.62
*x* ^2^ value		4.266	5.362
*P* value		0.014	0.023

**Table 5:** Multifactor logistic regression analysis of factors influencing postoperative incisional infection in two groups of patients.

Influence factor	*β* coefficient	Wald *x*^2^ value	*P* value	OR value	95% confidence interval
Operation time	1.705	18.744	0.002	6.587	0.837–1.273
Operation mode	2.328	14.325	0.005	15.730	0.764–1.057
Length of stay	1.509	16.099	0.004	5.710	0.780–0.982
Preoperative fever	1.337	17.394	0.003	5.998	0.879–1.259
Diabetes	2.427	22.029	0.001	17.881	0.739–1.154
Anemia	1.326	15.527	0.004	5.003	0.784–1.085

## Data Availability

The datasets used and analyzed during the current study are available from the corresponding author upon reasonable request.
